The article "Fog Computing Service in the Healthcare Monitoring System for Managing the Real-Time Notification" was published in 2022. Journal: J Healthc Eng.

# Fog Computing Service in the Healthcare Monitoring System for Managing the Real-Time Notification

**DOI:** 10.1155/2022/5337733

**Published:** 2022-03-15

**Authors:** Ahmed Elhadad, Fulayjan Alanazi, Ahmed I. Taloba, Amr Abozeid

**Affiliations:** ^1^Department of Computer Science, College of Science and Arts Qurayyat, Jouf University, Sakaka 72388, Saudi Arabia; ^2^Department of Computer Science, College of Computer and Information Sciences, Jouf University, Sakaka 72388, Saudi Arabia

## Abstract

A new computing paradigm that has been growing in computing systems is fog computing. In the healthcare industry, Internet of Things (IoT) driven fog computing is being developed to speed up the services for the general public and save billions of lives. This new computing platform, based on the fog computing paradigm, may reduce latency when transmitting and communicating signals with faraway servers, allowing medical services to be delivered more quickly in both spatial and temporal dimensions. One of the necessary qualities of computing systems that can enable the completion of healthcare operations is latency reduction. Fog computing can provide reduced latency when compared to cloud computing due to the use of only low-end computers, mobile phones, and personal devices in fog computing. In this paper, a new framework for healthcare monitoring for managing real-time notification based on fog computing has been proposed. The proposed system monitors the patient's body temperature, heart rate, and blood pressure values obtained from the sensors that are embedded into a wearable device and notifies the doctors or caregivers in real time if there occur any contradictions in the normal threshold value using the machine learning algorithms. The notification can also be set for the patients to alert them about the periodical medications or diet to be maintained by the patients. The cloud layer stores the big data into the cloud for future references for the hospitals and the researchers.

## 1. Introduction

Cloud computing provides a variety of IoT services, including computation resources, storage capacities, heterogeneity, and high processing that have accompanied a technological revolution. At many levels, the cloud allows for the virtualization of computational resources. Almost every aspect of human life has embraced cloud computing. Cloud computing, on the other hand, has limitations in terms of large delays, which have a negative impact on IoT jobs that demand a real-time reaction. It also does not work with industrial control systems that require a quick response time [1].

A concept of fog computing has been introduced to link IoT devices with data centers. Similar to IoT, fog computing has several applications like monitoring and analysis of data from network-connected things in real time and facilitates further actions to be taken. Fog computing is more virtualized and it can provide networking services among end devices and cloud computing data centers, but it is not entirely positioned at the edge of the network. Fog computing can be used at three levels of networking: (1) data collection from edge devices (sensors, vehicles, roadways, and ships), (2) multiple devices connecting to a network and sending all data, and (3) the collected data from the devices that should be processed in less than a second, along with decision-making [2, 3].

The article "Fog Computing Service in the Healthcare Monitoring System for Managing the Real-Time Notification" was published in 2022. Journal: J Healthc Eng.

The IoT is considered as a dynamic global network infrastructure, in which the things with unique characteristics are unified to enable advanced services. One of the basic technologies used in IoT healthcare is the Wireless Body Area Networks (WBANs). It can acquire the signals like body temperature, electrocardiogram (ECG), electromyography (EMG), and blood pressure. These data are transmitted to the end-users through the protocols like Wi-Fi or IEEE.802.15.4 for diagnosis and visualization. In healthcare monitoring, the remote cloud servers are in use to process and store the data from sensor nodes using cloud computing. But there are some challenges like latency sensitivity, large data transmission, and location awareness. Fog computing brings cloud capabilities closer to end-users by delivering storage, processing, and communication to edge devices, which improve mobility, privacy, security, low latency, and network bandwidth. Fog computing can ideally match latency-sensitive or real-time applications [4].

Real-Time Environmental Monitoring, Visualization, and Notification systems are considered to facilitate a new perspective in reliable data capturing, effective visualization, and handling emergency time-sensitive circumstances for Health and Safety management [5, 6]. In recent years, the population of aged people all over the world is increasing and hence complex health issues are also increasing which leads to increased clinical expenses. Remote health monitoring is vital for individuals, especially for the aged. This can help in reducing the additional expenses to be spent on hospitals. But the traditional models of healthcare monitoring are not so convenient and involve time-consuming processes. Hence, there is a demand for developing an efficient healthcare monitoring system that reduces the hospitalization of patients and also enhances the quality of life of the patients [7]. In the era of IoT, a huge amount of data is to be handled each and every second from several devices. Currently, cloud computing is used to handle such data. But the requirement of data centers which are highly expensive makes cloud computing infeasible for data processing, because of the larger distance between the data center and the sensing devices. As the healthcare data should be transmitted without any delay so as to get the proper response on time, fog computing is introduced in the field of health monitoring to improve the Quality-of-Service (QoS) [8].

The article "Fog Computing Service in the Healthcare Monitoring System for Managing the Real-Time Notification" was published in 2022. Journal: J Healthc Eng.

Mobile health (m-health) denotes the use of mobiles or smartphones in the collection of healthcare data from the patients in real time and storing them into a cloud server using the Internet. The hospitals, insurance providers, etc. can be able to access these data from the cloud so as to give proper treatment for the patients. The availability of wearable devices and body sensor networks helps in the invention of the m-health system. Integrating m-health in a patient's environment helps in real-time analysis of the patient's health [9]. For several healthcare applications, the use of a simple sensor-to-cloud system is not feasible due to the security concern and the issue of network failure that risks the patient's health due to the delay in accessing the patient data. Using only the cloud platform for healthcare data to be processed and stored results in the delay of transmitting the data from sensors to the cloud and from the cloud to hospitals. Hence, the use of fog computing is introduced in healthcare applications in situations that require emergency responses and real-time actions [10]. The number of patients using Implantable Cardioverter Defibrillators is going on to increase. It collects the data such as device functioning and physiological parameters so as to improve the survival of the patients. Monitoring those data in real time remotely helps in the early detection of clinical factors and promotes therapy adjustments or reprogramming the devices before the patients are hospitalized. Remote monitoring of health is highly effective compared to the traditional one-on-one consultation since it is highly reliable, safe, cost-efficient, and quick responsive regarding any failures, minimizes the hospital appointments, and reduces the unwanted shocks regarding their health condition [11].

The applications of IoT paves a way for the implementation of ambient-assisted living systems for providing assistance in health monitoring and even in the day-to-day activities of an individual. The patients monitored in hospitals, especially in Intensive Care Units (ICUs) by medical assistants sometimes, causes errors since the errors are inevitable for humans. Hence, it is essential to develop an IoT-enabled health monitoring system for patients needing permanent support, in any case, to accurately collect the health parameters to provide the right clinical support on time and to prevent unnecessary costs and efforts on improper monitoring [12]. Fog computing is formed by extending cloud computing to the edge of the network. Fog computing is not a substitute for cloud computing, but it will act as a complement to it. The heavy network traffic nowadays causes a huge burden in bandwidth while transmitting a large amount of data to the cloud, unbearable latency, and degraded services to the end-users. Hence, it is important to redesign the computing patterns so as to meet the necessities of the big data era [13]. A detailed systematic literature survey has been given in [14] which includes the motivations, limitations, and future recommendations in this field of IoT healthcare systems using fog computing. This survey describes that fog computing can be well suited for real-time applications that require high response time and low latency. It is clear from this review that fog computing decreases the latency compared to cloud computing, which is very much essential in the field of healthcare in real time.

The article "Fog Computing Service in the Healthcare Monitoring System for Managing the Real-Time Notification" was published in 2022. Journal: J Healthc Eng.

The objectives of the proposed fog computing paradigm are as follows: it may reduce latency when transmitting and communicating signals with faraway servers, allowing medical services to be delivered more quickly in both spatial and temporal dimensions. As a result, machine learning is used to process the data, which then becomes the outcome of interpretation. The proposed tools and technologies are explained in detail, including how they can work in tough circumstances and how they can be implemented in areas where IoT-driven healthcare services are most required. The rest of the paper is organized as follows: Section 2 presents related works undergone during the research process, Section 3 presents the proposed methodology, Section 4 gives results and discussion followed by Section 5 with a conclusion, and finally, the reference paper used in this research has been listed out under reference section.

## 2. Related Work

An IoT-based healthcare system that uses the fog computing concept is given in [4]. The efficiency of using fog computing in the field of health monitoring has been demonstrated based on the use of bandwidth, QoS, and notification alerts. Also, a case study on using ECG features extracted from the clinical data at the edge of the network in the implementation process has been given at last. This paper collects the data such as temperature, the humidity of surroundings, location of the patients, SpO2, Electro Encephalography (EEG), ECG, and EMG, and these data are transmitted using the communication protocols, namely, Wi-Fi, Bluetooth, ZigBee, or 6LoWPAN. The advancement in technologies allows significant use of wearable devices in the field of healthcare to be deployed with IoT. Instead of using external sensors for monitoring, the use of devices that are employed in an individual's day-to-day activities is encouraged, for example, mobile phones. Since mobile phones are devices that have various sensors built-in, like gyro meter, heartbeat sensor, accelerometer, etc., remote monitoring of patients can be supported only by using the mobile phones themselves. But the use of fog computing is necessary so as to facilitate computing, networking, and cloud data storing [15]. The security breaches include impersonation, data breaches, data integrity, eavesdropping, and collusion. The clinical data obtained from the sensors or IoT devices are highly susceptible to security threats. These data would be highly confidential and should be accessed only by authorized individuals. The security breaches make those data to be accessed by unauthorized individuals revealing its confidentiality. Hence, a solution for solving the security breaches in healthcare IoT systems has been given in [16], which provides a fog-based decentralized healthcare architecture with multiple virtual machines having the fog nodes distributed geographically for data management and processing. Each virtual machine is responsible for a specific type of data and request.

The article "Fog Computing Service in the Healthcare Monitoring System for Managing the Real-Time Notification" was published in 2022. Journal: J Healthc Eng.

A framework on Resource Preservation Net for systems in the emergency department using Petri net has been developed combined with custom cloud computing and edge computing technologies. The Resource Preservation Net is well suited for real-time applications in which the patient's length of stay (LoS), average waiting time, and resource utilization are considered vital performance indicators. Hence, in this framework, it is indicated that the LoS, average waiting time, and resource utilization are considerably improved [17]. The IoT concept which is the combination of sensors, smart devices, and the Internet and the middleware concept which is the combination of sensors and IoT devices have been described in [18]. This paper suggests that there will be a crucial motivation for the integration of middleware in e-health systems. The integration of middleware platforms in e-health systems is to improve the process of monitoring the general health of a patient or an individual. On-site research on IoT-based mobile medical information systems has been described in [19]. This research includes a questionnaire survey, evaluation of people's opinions which includes the disease diagnosis by hospitals, the treatments and the cost of treatment procedures, and hospital's information systems. With the help of the results obtained from the survey, the requirement analysis and design of the mobile medical information system had been accomplished.

The article "Fog Computing Service in the Healthcare Monitoring System for Managing the Real-Time Notification" was published in 2022. Journal: J Healthc Eng.

E-health and m-health provide hospitals, students, healthcare professionals, and researchers with various services like disease diagnosis, risk prediction, treatment analysis, health monitoring, education, and machine learning model development. In [20], a literature survey of the effective use of IoT in the healthcare domain has been carried out, followed by the development of a semantic model of e-health and named “k-Healthcare” for accessing the healthcare data by the patients effectively using smartphones. Since most of the existing e-health and m-health models do not use smartphone sensors for sensing and transmitting health data, the k-healthcare uses smartphones for sensing and transmitting the data shown in Figure 1. It consists of four layers of architecture, namely, the sensor layer, network layer, Internet layer, and finally a service layer. Each layer provides unique functions to facilitate efficient services to adjacent layers. A case study on the challenges faced in IoT because the models being limited to data centers cannot satisfy the needs of several IoT applications is given in [21]. This study focuses on 3 requirements such as mobility, actuation, and control of reliability and scalability, particularly where a large span of areas is covered and for real-time decision-making scenarios. The method of applying IoT, cloud computing, and fog computing in home-based hospitalization has been given in [22]. In addition to this, this paper also describes the concept of edge computing in remote health monitoring of patients and telehealth which supports the communication between healthcare professionals or doctors and the patients. This study indicates that the integration of fog computing and cloud computing in IoT healthcare technology provides quality services to patients. This method also proves that it offers high safety, reliability, and cost-effectiveness.

An IoT-based e-health system using fog computing offers patient-centric healthcare instead of clinic-centric treatment in which all authorities like patients, hospitals, and services are interconnected with each other seamlessly. The promises and the challenges faced during the transition of clinic-centric to patient-centric approaches have been demonstrated and described in [23]. This study described the benefits of applying IoT technology in e-health systems, which are as follows: all-encompassing, which means that it can be applied for different types of purposes like healthcare, exercising, beauty, safety, etc.; integrating with distinct technologies irrespective of its complexity seamlessly; analysis and processing of big data; personalizing the services; for instance, it can foresee and predict the health issues that would be caused in future so as to make the patients take necessary steps for prevention or curing; lifetime monitoring; easy to use; reduced cost; accessible at anywhere and anytime; more number of doctors could be involved if needed; online assistance; and better efficiency and international collaboration. A fog-centric smart home-based patient health monitoring system using IoT is demonstrated in [24]. The major objective of this system is to monitor the patients who need intensive care in their home itself remotely. This model consists of 5 layers, namely, data acquisition, event classification, information mining, decision-making, and cloud storage layers. Each layer is responsible for unique functions so as to provide better services to the adjacent layers. This paper offers services like home-based patient monitoring, event classification using fog computing to provide real-time response, temporal mining of health-related data from patients based on event triggering in the cloud layer, and real-time notification-based decision-making and data transmission to caregivers and hospitals in patient's unsafe conditions. A fog assisted Wearable IoT (wIoT) system for end-to-end analytics has been implemented in [25]. The fog computing can help getting efficient wIoT system. The wIoT devices are connected in one end and the cloud at the other end. In this paper, a prototype made of a middle layer, which is the smart for gateway using Intel Edison and Raspberry pi, has been developed. This prototype is designed to support data conditioning, filtering, analysis, and transmitting appropriate data to cloud for storing it for a long time and temporal variability monitoring. This prototype was tested with smart e-textile gloves system and observed that the conversion of real-world data to useful analytics with the help of knowledge-based models increases the usability of this system. Hence, it can provide better end-to-end interaction of wearables and cloud [26–29].

The article "Fog Computing Service in the Healthcare Monitoring System for Managing the Real-Time Notification" was published in 2022. Journal: J Healthc Eng.

## 3. Preliminaries

### 3.1. Fog Computing

Fog computing lies between the devices and cloud computing. This is made possible by introducing a new processing unit between the cloud and the user to enhance reliability, energy efficiency, and privacy maintenance and reduce latency. In addition to the advantages of cloud computing, fog computing also facilitates computing power, networking capability, storage capacity, and real-time data analysis. Fog computing also facilitates real-time notification systems on users' devices. Unlike cloud computing, fog computing reaches the users in no time, but latency is the main issue in cloud computing. But the fog computing is not as much powerful as cloud computing, since it makes use of low-end computers, mobile phones, and personal devices only.

The data from all devices have been transmitted to the fog computing devices which then go via various layers such as (1) Data Center/Cloud layer, (2) Core Domain/Network layer, (3) as Edge Domain layer, (4) Smart Sensors layer, and finally, (5) Smart Monitoring layer as given in Figure 2. To overcome data corruption, a security layer exists between the end-user device and the computing devices. The data are then transmitted to the devices of fog computing for processing. This step is called preprocessing. These data are not big data. Only a small amount of data will get processed by fog computing devices. An additional advantage of fog computing is that there is a temporary storage layer that can store the processed data, which can be sent later to cloud computing for processing further.

The maintenance of a fog computing network will be highly complicated. The maintenance persons will take care of the network if there occurs any fault in the network during data transmission. The major advantage is the fact that the computational service could learn and adapt the possible outcomes obtained from fog computing.

### 3.2. Fog Computing in Health Monitoring

Fog computing is a novel standard in the system of healthcare monitoring. Fog computing facilitates data processing without reducing its quantity and also prevents network congestion. The remote healthcare system makes use of body sensors that are embedded into the patient body or perfectly positioned on the body to monitor the health status of the patients by gauging certain signs and to assist them in getting exact solutions. A specific device is used in collecting the data from those body sensors and also supports the communication between the sensors and the monitoring devices.

## 4. Proposed Methodology

Healthcare issues are becoming more prevalent in overpopulated countries, such as India, as the population grows and the need for medical assistance grows. The population's need for high-quality care is increasing, while treatment costs are decreasing. Technology has progressed to the point that health can be monitored remotely via a machine, which is more dependable than manual monitoring. It can assist in reducing the time spent on individual personal training and increasing the reliability of advanced machinery. Wearable devices, which track everything and everyone in every imaginable way, are one form of fog computing that is disrupting our day-to-day lives on a daily basis. The devices, which are wearable by people, contain a variety of sensors. These devices maintain track of a variety of human activities. Wearable devices provide a new edge for healthcare, but the potential of the Internet of Things is growing in every discipline, not just medical sciences. These wearable devices make life easier and more comfortable for people by tracking health data, as well as safety and security and their associated technologies.

The article "Fog Computing Service in the Healthcare Monitoring System for Managing the Real-Time Notification" was published in 2022. Journal: J Healthc Eng.

There is an existing system for triparty, one-round key authenticated agreement, employing fog computing facilities, and it used bilinear pairing encryption to generate a session key between the persons to assure safe communication. A new computational framework for remote real-time monitoring, sensing, and scaling high-performance computing for prognosis and diagnosis has been proposed in this paper.

The proposed healthcare monitoring framework consists of three layers, namely, (1) sensor network layer, (2) fog layer, and (3) cloud layer. The architecture of the proposed fog-based health monitoring framework is given in Figure 3. These layers are described as follows.

### 4.1. Sensor Network Layer

In order to sense the temperature, pulse rate, and blood pressure of a patient, sensors such as temperature sensor, ECG sensor, and blood pressure sensor are used along with a wearable device in which these sensors have been embedded so as to be comfortably worn by the patients. All these sensing devices form the sensor network layer. This layer senses the patient's health conditions which include the patient's body temperature, heart rate, and systolic and diastolic blood pressure and collects the data using the sensors. These data are then transmitted to the fog computing devices through wired or wireless communication protocols.

### 4.2. Fog Layer

The fog layer comprises several distributed nodes. These nodes are called gateways. The gateway is a device that facilitates storing, computing, and network connection that is distributed near the sensors. These sensors are responsible for recording the events and producing the data. This layer facilitates four operations: data reception from sensors, analysis of those data for health-related decision-making, notifying the caregivers, and storing all these data in the cloud. In order to improve the reliability of the system, reduce latency, prevent network connectivity issues, and increase the speed of decision-making processes, a local data processing system has been implemented in fog computing to improve its intelligence. The properties of the fog layer are given as follows:

- Data collection: the data from various sensors like temperature sensors, ECG sensors, and blood pressure sensors, which are connected to the wearable device, are collected for further analysis and decision-making process. After collecting the data, filtering, noise removal, and preprocessing are performed.
- Data security: the data of patients obtained from the sensors are to be transmitted from gateway devices to the cloud. Hence, there is a need for the security and integrity of such data to be considered in the design of a healthcare monitoring framework. Thus, a process of encryption and watermarking has been implemented so as to secure the proposed framework. In the encryption process, the data are converted to an unrecognized format so as to protect them from unauthorized persons. In the watermarking process, the data are hidden behind an image without any distortion in its credibility or visibility [30–34].
- In the proposed system, the patient's data are hidden under the patient's face image by watermarking while storing in the fog server or transmitting to the cloud server. After that, the watermarked image has been converted into a cipher image using an appropriate encryption algorithm. This encrypted data cannot be read by unauthorized persons. The data needs to be stored under the patient's image; this is done because the data cannot be opened unless permission is given by the authorized person. The data must be hidden because these data are used to be stolen and people improve their intelligence in blackmailing by these collected data.  Figure 4 shows the process of watermarking and encryption of data into a face image. Meanwhile, the author states that the storage space is a concern and thus it is necessary to compress the data. The transmission of the patient's image for each collected data turns out to be an excessive overheard. By adjusting the parameters in the model and changing the evolution mechanism of the network, the robustness of fog computing can be improved.
- With this growth, fog computing scale with its related edge computing paradigms, such as multiaccess edge computing and cloudlet, is seen as promising solutions for handling the large volume of security-critical and time-sensitive data that is being produced by the IoT.
- Local storage*:* there will be a local storage in the gateway which serves as a local repository for storing the data for analysis and security processing. In addition to this, the data will be stored temporarily in the local storage before transmission, and even if there occurs a network cut-off, the data will be temporarily stored there till the network is resumed.
- Notification service*:* the notification system sends notifications in tough situations of patients to the doctors or caregivers. Notification can also be sent to the patients to take proper medication on time or alerting their food time and what to eat and some other instructions to be followed by the patients.
- Data analysis: the data collected from the temperature, ECG, and blood pressure sensors are stored in the fog layer, where they are analyzed for any emergency situations based on age, height, weight, and disease using a machine learning approach. If this analysis shows any contradictory situation, then a notification will be sent to the authorized persons and transmit the data through the cloud. If the analyzed data is normal, then no action will be taken further, and no data will get transmitted.
- Data compression: the patient's data obtained from several sensors are stored in the cloud storage. These data could be used for disease prediction, risk analysis, and long-term use for researchers. Hence, a large amount of data would be stored in the cloud which makes the network congested, increases latency, and needs more storage space. Data compression is the best way to solve such a problem. There are two types of compression available: lossless compression and lossy compression. The proposed system uses lossless compression since the loss in medical images gives distortions in the data and leads to improper diagnosis of diseases and risk predictions. The lossless compression involves two steps which include changing the format of the image and then removing coding redundancy using an entropy encoder.

The article "Fog Computing Service in the Healthcare Monitoring System for Managing the Real-Time Notification" was published in 2022. Journal: J Healthc Eng.

### 4.3. Cloud Layer

The cloud layer is composed of the distributed resources, the repositories, and the servers. The cloud manager is responsible for managing all the devices connected to the cloud layer and facilitates the patient's data reception, processing, and storing. These data can be used for analyzing the patient's health history and current status. The properties of the cloud layer are given as follows:

- Data storage*:* after the process of data analysis of the fog layer, the analyzed data are transmitted to the cloud layer, which provides a large storage space for storing the patient healthcare data for future analysis for caregivers, doctors, hospitals, and insurance providers.
- Data analysis*:* the patient's health data, which includes the images of diseased parts, details of symptoms, treatments, and therapy plans, stored in the cloud, are subjected to analysis for future research purposes in the field of clinical decision-making. Several machine learning approaches and data visualization techniques could be implemented so as to obtain more understanding from these data.
- Disease prediction*:* the possibility of which disease the patient will get affected in the future can be predicted by the age, height, weight, and patient's hereditary. With respect to the correlation of the vital signs, the percentage of disease expectation can be predicted by using machine learning Algorithm 1.

The article "Fog Computing Service in the Healthcare Monitoring System for Managing the Real-Time Notification" was published in 2022. Journal: J Healthc Eng.

## 5. Discussion

The data flow of the proposed health monitoring framework is given in Figure 5.

- The data from sensors are collected and are subjected to analysis.
- The unwanted noise, electromagnetic interferences, and inappropriate attachments of sensors are filtered. The filtered data are analyzed so as to diagnose the current health situation of the patient.
- After data analysis, if any contradictions are found in the sensed health parameter values, then a notification will be sent to the doctors or caregivers of the patients who are in need of assistance regarding their health status.
- The data collected and processed are allowed to be stored in the cloud for accessing them in the future for researchers, healthcare professionals, or the patients if needed. The stored data will be watermarked under the patient's image and are encrypted to preserve the security of the patient's data during transmission and storing.
- These data are compressed so as to minimize the storage space required since, in the big data era, storage space is a high concern.
- The data are temporarily stored locally in the fog, in case of any network failure occurs.
- The most common way of getting data out of smart sensors is to use a bridging device known as a gateway in each room. A gateway receives data from the sensors and makes it useable. Data is transmitted from the sensors to the gateway wirelessly.
- A smart electrical grid is a use case for fog computing. In order to function efficiently, smart cities must respond to rising and falling demands, reducing production as needed to stay cost-effective. This means that smart grids demand real-time electrical consumption and production data.
- Fog computing works by utilizing local devices termed fog nodes and edge devices. Raw data is captured by IoT beacons. This data is sent to a fog node close to the data source. This data is analyzed locally, filtered, and then sent to the cloud for long-term storage if necessary.

For IoT designers, fog computing serves as the best choice due to its following features:

- fog computing can provide better delay performance since the position of fog resources will be between the smart devices and the cloud data centers.
- fog computing requires micro centers with limited processing, communication, and storage facilities; the cost of distribution of micro fog centers near the end-users will be very less when compared to the cloud data centers.
- The IoT systems are highly scalable in fog computing, which means that if the end-user increases, the micro fog centers could also be deployed more to compensate for the increase in load. The increase in the deployment of the cloud data center is not much possible, since the cost will be very high.
- Fog computing provides replicated and robust services.
- The fog resources can serve as mobile cloud since the fog resources are deployed closely with the end-users.
- The real-time services can achieve high performance with fog computing.
- The fog resources can be interoperable with several cloud service providers. Hence, fog computing and its resources are highly standardized.
- Data aggregation can be performed by fog resources for sending the data that are processed partially as an opposition with the raw data to cloud data centers for processing it further.

The article "Fog Computing Service in the Healthcare Monitoring System for Managing the Real-Time Notification" was published in 2022. Journal: J Healthc Eng.

Hence, it is evidenced that fog computing has the ability to enhance the IoT device performances since a part of high-level services provided by cloud computing can be performed by local resources.

## 6. Evaluation

Test results on the customized ECG equipment were performed during the sample assessment processes with various functioning conditions, including sampling rates and channel count. The number of stations must be between 6 and 12, as well as the sample rate must be between 550 Hz and 1 kHz. The data for the longest recorded duration utilizing the software's embedded 4 GB NAND Flash Storage are summarized in Table 1. In both operating conditions, as indicated in Table 2, the duration of the devices in terms of capacity charge is also examined, in particularly the real resource usage of the most precise sampling frequency of 1 kHz for 12 channels.

The Android Applications were assessed by determining the overall storage space required to store an ECG tracing with several channels and two different sampling speeds (1 kHz and 550 Hz) in EDF + formats. The entire period of all ECG traces was one minute. It is feasible to reduce the storage amount required by using compression technologies, but this would have an instant impact on battery capacity. In two different settings, the data communication rate of the ECG equipment was also tested as illustrated in Table 3.

The wearable ECG equipment could send information to a mobile phone in two modes: downloads mode, which sends information from the ECG software's memory, and monitoring mode, which sends data from the present recording in real time. The wearable ECG equipment could be in either an inactive or active recording phase when there is data transmission from an ECG. In the latter instance, the technology of the wearable ECG equipment restricts the information transfer rates to the mobile phone in order to maintain the efficiency of the active recorded collecting data.

The article "Fog Computing Service in the Healthcare Monitoring System for Managing the Real-Time Notification" was published in 2022. Journal: J Healthc Eng.

The information transfer rates also differ depending on whether the ECG equipment saves the information when transferring it or if the information is delivered straight without being stored in the internal storage. The transmission of data occurs in the first scenario after the information is recorded in the storage (each admission in the storage occurs only after a full information site has been loaded), and the data is read from their saved location to establish transmission packages with a predetermined number of samples described by the device software. In the second scenario, data transfer occurs immediately after the ADC inverters have sampled the data and acquired a predetermined number of samples. The sampling frequency, the number of channels employed in the recorder, and the preset maximum number of transfers each second are used to determine the predetermined packets for information transfer.

Tables 4 and 5 illustrate the information read rates from the ECG equipment to the mobile applications for various ECG device setups, as measured by the mobile phones. We should point out that we not only transfer and measure information packets during transmitting data but also regulate and acknowledge packets, energy capacity phase report packets, and reconnection packets (in the event of a separation). These packets are frequently transmitted, but they can have an impact on the theoretically possible throughput in the communications among the ECG and the cellphone.

Any authorized users with accessibility to the Spark-Heart prototype's online site, which is accessible via the clouds, can send instructions to the Smartphone Applications and Wearable Gadgets, which pass through the system's specific interfaces. We estimated the maximum and average response time of simple condition demands (for example, ECG trace counts, remaining memory, and battery level) toward the ECG machine, as well as the maximum and average time the structure takes to make a problem for a full document of the existing ECG device state, to evaluate the end-to-end response time of such a request.  Table 6 presents a summary of the results.

## 7. Conclusion

This paper proposed a fog-based health monitoring framework, which makes use of fog gateways for clinical decision-making based on the data collected from the sensors like temperature sensor, ECG sensor, and blood pressure sensor, which are embedded into a wearable device so as to measure the temperature, heart rate, and systolic and diastolic pressure of a patient. These data are then secured by watermarking and encryption processes and are temporarily stored in the fog server until receiving proper network connectivity and transmitting them to the doctors or caregivers via the cloud in case of any emergency situations. This increases the utility of the proposed system. The huge amount of data collected from these sensors is compressed and stored in the cloud server for future references of hospitals and researchers. Finally, in this paper, the benefits of choosing fog computing services in healthcare monitoring and clinical decision-making have been discussed.

The article "Fog Computing Service in the Healthcare Monitoring System for Managing the Real-Time Notification" was published in 2022. Journal: J Healthc Eng.

## Figures and Tables

**Figure 1:** Fog distributions to end-users by cloud.

**Figure 2:** Various layers of fog computing.

**Figure 3:** Architecture of the fog-based health monitoring framework.

**Figure 4:** Watermarking and encryption process.

**Figure 5:** Flow diagram for the proposed system.

**Algorithm 1:** Predicting patient health status and notifying the authorities.

**Table 1:** Maximum length of recording.

Sample range (kHz)	Channels	Duration (hrs)
1	6	59.73
550	6	120.53
1	12	30.91
550	12	15.10

**Table 2:** Maximum operation lifetime.

Operation	Channels	Sampling rate (kHz)	Device lifetime (hrs)
Real-time data transfer	12	1	7.51
Non-real-time data transfer	12	1	19.62

**Table 3:** ECG trace parameters.

Channels	Sampling rate (kHz)	Total size (KB)
6	550	376.525
6	1	735.4
12	550	1.506
12	1	735.4

**Table 4:** Direct transmission of an ECG trace.

Channels	Sample rate (kHz)	Average throughput (kbps)	Storing memory
6	550	11.620	Yes
6	550	15.379	No
6	1	22.929	Yes
6	1	27.083	No
12	550	36.844	Yes
12	550	47.544	No
12	1	76.099	Yes
12	1	97.699	No

**Table 5:** ECG transmission storage.

Channels	Sample rate (kHz)	Average throughput	Sampling
6	550	13.158 kbps	Yes
6	550	1.566 Mbps	No
12	1	78.665 kbps	Yes
12	1	640.198 kbps	No

**Table 6:** Response time maximums and averages.

Command type	Maximum response (ms)	Average response (ms)
Simple report	49.829847	22.499428
Completed report	139.450269	107.994685

## Data Availability

The data used to support the findings of this study are included within the article.

## References

[1] Mani N., Singh A., Nimmagadda S. L. (2020). An IoT guided healthcare monitoring system for managing real-time notifications by fog computing services. *Procedia Computer Science*.

[2] Nandyala C. S., Kim H.-K. (2016). From cloud to fog and IoT-based real-time U-healthcare monitoring for smart homes and hospitals. *International Journal of Smart Home*.

The article "Fog Computing Service in the Healthcare Monitoring System for Managing the Real-Time Notification" was published in 2022. Journal: J Healthc Eng.

[3] Taloba A. I., Alanazi R., Shahin O. R., Elhadad A., Abozeid A., Abd El-Aziz R. M (2021). Machine algorithm for heartbeat monitoring and arrhythmia detection based on ECG systems. *Computational Intelligence and Neuroscience*.

[4] Gia T. N., Jiang M., Rahmani A.-M., Westerlud T., Liljeberg P. Fog computing in healthcare internet of things: A case study on ecg feature extraction.

[5] Kiani A., Salman A., Riaz Z. (2014). Real-time environmental monitoring, visualization, and notification system for construction H&S management. *Journal of Information Technology in Construction*.

[6] Alanazi F., Elhadad A., Hamad S., Ghareeb A. (2019). Sensors data collection framework using mobile identification with secure data sharing model. *International Journal of Electrical and Computer Engineering*.

[7] Nguyen H. H., Mirza F., Naeem M. A., Nguyen M. A review on IoT healthcare monitoring applications and a vision for transforming sensor data into real-time clinical feedback.

[8] Al-Khafajiy M., Webster L., Baker T., Waraich A. Towards fog driven IoT healthcare: challenges and framework of fog computing in healthcare.

[9] Almotiri S. H., Khan M. A., Alghamdi M. A. Mobile health (m-health) system in the context of IoT.

[10] Paul A., Pinjari H., Hong W.-H., Seo H. C., Rho S. (2018). Fog computing-based IoT for health monitoring system. *Journal of Sensors*.

[11] Bertini M., Marcantoni L., Toselli T., Ferrari R. (2016). Remote monitoring of implantable devices: should we continue to ignore it?. *International Journal of Cardiology*.

[12] Chiuchisan I., Costin H.-N., Geman O. Adopting the internet of things technologies in health care systems.

[13] Deng R., Lu R., Lai C., Luan T. H. Towards power consumption-delay tradeoff by workload allocation in cloud-fog computing.

[14] Mutlag A. A., Abd Ghani M. K., Arunkumar N., Mohammed M. A., Mohd O. (2019). Enabling technologies for fog computing in healthcare IoT systems. *Future Generation Computer Systems*.

[15] George A., Dhanasekaran H., Chittiappa J. P., Challagundla L. A., Nikkam S. S. Internet of Things in health care using fog computing.

[16] Awaisi K. S., Hussain S., Ahmed M., Khan A. A., Ahmed G. (2020). Leveraging IoT and fog computing in healthcare systems. *IEEE Internet of Things Magazine*.

[17] Oueida S., Kotb Y., Aloqaily M., Jararweh Y., Baker T. (2018). An edge computing based smart healthcare framework for resource management. *Sensors*.

[18] dos Santos A. P., Lima D. W. S., Freitas F. S., da Silva G. M. A motivational study regarding IoT and middleware for health systems.

[19] Sun G., Yu F., Lei X., Wang Y., Hu H. “Research on mobile intelligent medical information system based on the internet of things technology.

The article "Fog Computing Service in the Healthcare Monitoring System for Managing the Real-Time Notification" was published in 2022. Journal: J Healthc Eng.

[20] Ullah K., Shah M. A., Zhang S. Effective ways to use Internet of Things in the field of medical and smart health care.

[21] Yannuzzi M., Milito R., Serral-Gracià R., Montero D., Nemirovsky M. Key ingredients in an IoT recipe: Fog computing, cloud computing, and more fog computing.

[22] Ijaz M., Li G., Lin L., Cheikhrouhou O., Hamam H., Noor A. (2021). Integration and applications of fog computing and cloud computing based on the internet of things for Provision of healthcare services at home. *Electronics*.

[23] Farahani B., Firouzi F., Chang V., Badaroglu M., Constant N., Mankodiya K. (2018). Towards fog-driven IoT eHealth: promises and challenges of IoT in medicine and healthcare. *Future Generation Computer Systems*.

[24] Verma P., Sood S. K. (2018). Fog assisted-IoT enabled patient health monitoring in smart homes. *IEEE Internet of Things Journal*.

[25] Constant N., Borthakur D., Abtahi M., Dubey H., Mankodiya K. Fog-assisted wiot: A smart fog gateway for end-to-end analytics in wearable internet of things.

[26] Al-Mashhadani R., Alkawsi G., Baashar Y., Ahmed Alkahtani A., Hani Nordin F. (2021). Deep learning methods for solar fault detection and classification: A review. *Information Sciences Letters*.

[27] Al-Sammarraee A., Alshareeda N. J. I. S. L. (2021). The role of artificial intelligence by using automatic accounting information system in supporting the quality of financial statement. *Information Sciences Letters*.

[28] Atia I., L Salem M., Elkholy A., Elmashad W., Am Ali G. J. I. S. L. (2021). In-silico analysis of protein receptors contributing to SARS-COV-2 high Infectivity. *Information Sciences Letters*.

[29] Al-Rawi Y. M., Al-Dayyeni W. S., Reda I. J. I. S. L. (2021). COVID-19 impact on education and work in the kingdom of bahrain: survey study. *Information Sciences Letters*.

[30] Sengan S., Khalaf O. I., Vidya Sagar D. K., Sharma D. K., Prabhu Q. A. J., Hamad A. A. (2022). Secured and privacy-based IDS for healthcare systems on E-medical data using machine learning approach. *International Journal of Reliable and Quality E-Healthcare*.

[31] Syed S. A., Sheela Sobana Rani K., Mohammad G. B., Chennam K. K., Jaikumar R. (2022). Design of resources allocation in 6G cybertwin technology using the fuzzy neuro model in healthcare systems. *Journal of Healthcare Engineering*.

[32] Karar M. E., Al-Rasheed M. F., Al-Rasheed A. F., Reyad O. (2021). IoT and neural network-based water pumping control system for smart Irrigation. *Information Sciences Letters*.

[33] Ammer S. M. E. I. (2021). Content analysis of lighting and color in the embodiment of fear concept in horror movies: a Semiotic approach. *Information Sciences Letters*.

The article "Fog Computing Service in the Healthcare Monitoring System for Managing the Real-Time Notification" was published in 2022. Journal: J Healthc Eng.

[34] Karar M. E., Alotaibi F., Rasheed A. A., Reyad O. (2021). A pilot study of smart agricultural irrigation using unmanned aerial vehicles and IoT-based cloud system. *Information Sciences Letters*.

